The article "Analysis on the Development and Influence of National Fitness Environment on Youth Basketball Coordination and Mental Health" was retracted in 2023. Reasons: signs of a paper mill; suspected computer-generated content; unreliable results or conclusions; concerns about the data.

# Analysis on the Development and Influence of National Fitness Environment on Youth Basketball Coordination and Mental Health

**DOI:** 10.1155/2022/6340347

**Published:** 2022-07-31

**Authors:** Pengfei Lu, Yajuan Su

**Affiliations:** ^1^Nanyang Normal University, Institute of Physical Culture, Nanyang 473000, China; ^2^Nanyang Institute of Technology, Physical Education Department, Nanyang 473000, China

## Abstract

In order to improve the basketball theory and provide theoretical and intellectual support for the scientific, mental health, and sustainable development of basketball, we propose to take the development dynamic mechanism of juvenile basketball as the research object and make a systematic and in-depth study on the dynamic mechanism, the cultivation of Chinese and foreign juvenile basketball reserve talents, and the dynamic dilemma and influencing factors of juvenile campus basketball development by using the methods of literature, questionnaire, and expert interview. A method of cultivating the ring tone of juvenile basketball is proposed. This method is based on Chan algorithm. When the target is close to each base station, the first estimation also needs an initial value to solve the initial solution estimation matrix. The method is also based on multivariate Taylor algorithm, taking into account the measured distance between the targets to be measured, so it will get some useful information, which will improve the positioning accuracy. The experimental results show that the accuracy of the algorithm used in this paper is more than 85%. However, the accuracy of rebounding and passing recognition and prediction is low. The recognition accuracy and prediction accuracy of the test set are slightly lower than that of the effective set, which shows that the performance of the target detection system model in this paper can be further improved through more significant training examples. It is proved that the algorithm based on Taylor ring can meet the needs of teenagers in the basketball coordination and mental health.

## 1. Introduction

The development of national fitness has been more than 20 years, and national fitness has risen to the height of national strategy. Although there are many discussions on the issues related to national fitness, there are still deficiencies in theoretical research. Basketball has made brilliant achievements, but its position in the world and even in Asia has declined in recent years. The reason is that many contradictions between the theory and practice of basketball reserve talents, especially young basketball reserve talents, are becoming increasingly prominent, and there is a lack of motivation. As an innovative action with the characteristics and significance of the times, national fitness not only is prominently reflected in the development of mass sports, but also has become an important aspect that can continuously provide and improve the needs of sports fitness for all citizens and significantly improve the health quality of all citizens. In terms of developing productive forces, mobilizing the people to participate in sports activities is an investment that can return the maximum benefits. In terms of human needs, national fitness is consistent with the ultimate goal of socialism to enable people to live a happy, civilized, scientific, and healthy life. As the masters of society, the people should and can enjoy everything given to them by sports. In terms of social development, it should include the development of social undertakings such as science and technology, education, culture, health, and sports, as well as social employment, social security, social equity, and social harmony. Therefore, today's national fitness is not only a mass sports development plan, but also an idea, a direction, and a cause. It has become an operation symbol for coordinating all elements and aspects of mass sports to play a role in a certain direction. It has become a mechanism for coordinating the development process of mass sports and promoting the development of mass sports. At present, from the perspective of relevant domestic research, there is still little interpretation and analysis of the connotation of national fitness, mainly focusing on the current situation and existing problems of the use of national fitness path, the development and role of social instructors in national fitness, the current situation and countermeasures of national fitness, the research of national fitness service system, and the interpretation and analysis of relevant documents. Therefore, judging the connotation of national fitness from a theoretical perspective, breaking through the previous conventional research and using philosophical thinking to break the common sense is the direction of this paper, which will help to eliminate the current widespread one-sided and vague understanding of its concept, so as to lay a foundation for the research of national fitness-related issues. After visiting, introducing, and training in recent years, some parts of China are no stranger to functional physical training. Whether scholars engaged in physical training research or physical coaches practicing in the front line, their understanding of functional physical training tends to be complete and systematic, which has not only emerged a large number of scientific research achievements, but also made great contributions to the excellent achievements of national and provincial sports teams. However, in many underdeveloped areas, nonmain or youth sports teams are unfamiliar with functional physical training. Functional physical training should gradually spread from the spire of the “pyramid of Chinese competitive sports” to the middle and lower levels, so as to lay a solid foundation for Chinese competitive sports. In this new era of rapid development and ever-increasing challenges, in addition to heavy academic pressure, China's youth groups are also faced with complex changes in the social environment and interpersonal relationships. However, compared with college students and adults, the mental level and personality of most teenagers are still in a stage where they need to be properly guided and systematically cultivated and shaped, so when they encounter the above problems, they will inevitably experience anxiety, depression, emotional out-of-control, negative emotions such as conflict with others, self-defeating, and even more serious mental health problems, resulting in incorrect social behavior. In order to relieve and release the pressure of study and social life borne by young students, you can try to carry out a moderate amount of physical exercise, so as to release the pressure in a scientific way, adjust the psychological state, while relaxing the body, and finally achieve the purpose of learning and living happily.

## 2. Literature Review

Under the unified organization of the State General Administration of Sports, since 1996, China has gradually installed equipment for residents' fitness activities in urban communities and rural villages and towns. This project is known as the national fitness path project. In recent years, with the active promotion of the national fitness path, it has played a good role in promoting the development of urban community sports and fitness activities for urban residents. Huertas et al., in the evaluation of the awareness rate and use status of the national fitness path project, studied the three cities of *B*, *h,* and *C* by random sampling. The results show that the awareness rate of the path project in the urban community is high, the use of path equipment has a significant mood improvement effect, and the use of path equipment is safe [1]. Yao et al. applied the methods of literature reading, interview survey, questionnaire survey, and mathematical statistics in the article “Research on the Path Management System of National Fitness in C City under the Background of the Implementation of National Fitness Tiaoli.” Through the investigation of the number of existing fitness paths in various districts of Changsha, the following conclusions are drawn.

The reason for the damage of fitness path is the lack of maintenance, equipment, management, and guidance personnel, which is still the main contradiction hindering the development of national fitness path project in Changsha [2]. Al Hajaj et al., in the article “Research on the Necessity of Constructing the Insurance System of China's National Fitness Path Project,” focus on the national fitness path project, taking the fitness path management unit, exercise crowd, and fitness path equipment as the main body. This paper studies the degree to which sports insurance is needed in the field of national fitness path project. We put forward the concept of system construction and believe that the fitness path engineering insurance should keep up with the needs of the development of the times, establish the national health path engineering insurance system as soon as possible, timely and effectively solve the problems caused by sports injury accidents on the fitness path, and eliminate the worries of the majority of sports lovers [3]. The construction of the national fitness path project insurance system is a complex and systematic project, which requires us to think and study together, refer to the experience of foreign mass sports insurance system construction, and explore an insurance system suitable for the national fitness insurance system, so as to provide help for the development of the national fitness cause. In “Research on the Current Situation and Countermeasures of Rural Fitness Paths--Taking *Z* City as an example,” Samuel and Rastogi investigated and studied the construction, use, and management of rural fitness paths by using the research methods of literature, questionnaire, expert interview, and mathematical statistics. It was found that the types of rural fitness paths are relatively perfect and the layout is relative, but there are different degrees of losses, which need to be repaired and updated [4]. Rural users are mainly middle-aged and elderly people, and most of them exercise in the morning and evening, but they lack professional fitness methods and means. The utilization rate of rural fitness path is not high, and there is a lack of corresponding fitness guidance. It is necessary to establish relevant supervision and evaluation system. See Figure 1.

Abu Hussain, in the current situation investigation and countermeasures analysis of sports for the disabled in the implementation of the national fitness plan, through the methods of literature, questionnaire, interview, and mathematical statistics, conducted research from the aspects of the recognition of the disabled to the national fitness and the attitude, motivation, and way of participating in fitness activities [5]. The results show that the disabled hold a high positive attitude towards national fitness activities, but due to the constraints of internal and external factors, fitness has become an extravagant hope. Antonova used literature survey, questionnaire survey, GIS analysis, and social statistics as the main methods in the investigation and research on the current situation of the implementation of the national fitness project in *D* city. Through the investigation of residents and managers of community neighborhood committees in downtown *D* and based on the GIS platform of the national fitness project, the factors affecting the implementation of the national construction project are combined with the advantages of GIS technology to describe and analyze the status and effect of the implementation of the national fitness project in downtown *D* [6]. The results show that the number of women participating in fitness path exercise is more than that of men. There is little difference between the two. In terms of educational level, the number below junior middle school is the largest, and the number of participants is decreasing with the improvement of educational background. At present, the people participating in path fitness are middle-aged and elderly people. Most residents do not know the specific content of the national fitness project; that is, they are not yet aware of it. The layout of fitness facilities is an important factor affecting the implementation of the national fitness project, because population distribution and travel traffic have affected the utilization rate of fitness facilities. At present, the management of fitness path in each street community is insufficient, which directly leads to the occurrence of man-made destruction and theft. Traffic problems have also become the main influencing factors for community residents to participate in fitness activities. At present, the number and scale of community fitness paths in the central area of Dalian cannot meet the fitness needs of residents. See Figure 2.

From the perspective of the development of foreign basketball, although the process of basketball career in various countries continues to advance, there are great differences in social system, economy, politics, and development process in different countries, resulting in different development of competitive sports. The research on the development theory of campus basketball plays an important role in the competitive sports theory of various countries. With its continuous development, it has been enriched. Experts and scholars from various countries have made extensive and in-depth exploration on the development of campus basketball, made due contributions to the basketball competitive sports of various countries and constantly enriched the theoretical system of basketball.

Samuel and Rastogi pointed out in the article “Data Performance of Community Sports” that the core of the development power of modern campus basketball is the continuous injection of capital investment, and the capital investment channels should be diversified. A single national investment will lead to rigid operation mode, loss of flexibility, and reduced system operation efficiency [4]. The school should ensure the funds for basketball student athletes to participate in basketball activities, provide corresponding material rewards, ensure the activity participation rate of student athletes, and vigorously improve the mass base of school basketball, so as to continuously promote the benign development of campus basketball. Guseman et al. in the article “Ideal Tool for the Connection between Colleges and Universities and the Outside: Inter School Sports,” believed that the university has an important role in students' personal identity. Regular sports participation in high-level schools outside will also be an important tool for the university to obtain support [7]. Especially involving the coordinated development of external enrollment, alumni relations, community affairs, and government relations, the participation of college sports can promote the important development of various systems.

At the competitive level, Lan et al. pointed out in the research on the relative age effect of France young basketball players that for the long-term development of basketball, teenagers are an important part of campus basketball. For basketball, the cultivation of competitive talents needs to be distinguished at different ages, and about 7–12 years old is more suitable for the cultivation and development of competitive reserve talents [8].

Arede believes that whether youth campus sports can reach the ideal state depends on the will of the rulers and the position of sports in the national economy and national life at different time stages [9]. Therefore, its driving force mainly comes from the preference of the system, the judgment of policy makers, and the national sports values. The dynamic characteristics of all other cultural entities are similar in youth campus sports. The dynamic characteristics of youth campus sports have class hegemony, ideological deprivation, and the compulsion of operation principles. These characteristics have become the dynamic development symbol of youth sports development to a certain extent, but they are also the magic cube that restricts the development of youth sports. Therefore, the reform of youth campus sports power must release power, return government to the people, and develop moderately and freely. Pham and Hwang believes that the sports motivation and career performance of immigrant young football players are correlated with their foreign cultural adaptation. Athletes with strong foreign cultural adaptation and high cultural identity have a higher motivation foundation in sports, their continuous sports career is longer, and they may create better sports performance in their future sports career, so they have a higher probability of becoming excellent athletes [10]. Guseman et al. believe that among the many dynamic mechanism elements of teenagers' participation in sports, social support elements, family support elements, peer support elements, friend support elements, and coach support elements are very important [7]. The continuous and lasting input of these elements is an important weight for them to participate in the sport and achieve excellent results. Therefore, building a good social psychological support channel system to realize smooth and continuous psychological support input is the lubricant and booster to promote teenagers to participate in sports. See Figure 3.

Looking at the above research, although the relevant theoretical research results are rich and different perspectives, which reveals part of the reasons for the decline of the overall strength of competitive basketball to a certain extent, there are still some deficiencies in the following aspects. (1) There are many macro overall theories, and the research on micro operability is weak. Many studies tend to analyze the reasons for the weakness of the driving force of Chinese campus basketball from the macro system field, which makes the research like a castle in the air, with lack of foundation and too macro and micro operability, so that the research validity is weakened, and the popularization and effectiveness of the research results are not strong. (2) The transitional transplantation of foreign theories does not accord with the reality of China's system. Most of the existing studies cite the successful experience of developing teenagers' basketball into a powerful country. Although the development of teenagers' campus basketball in various countries has certain common laws to a certain extent, the process of education and social development in different countries has different characteristics [11]. China is in a period of dual track development. The dynamic factors of campus basketball development are complex and changeable. It is not embedded in the reality of China's system, which is not enough to reveal the most essential aspect of the dynamic dilemma of Chinese campus youth basketball development. Moreover, the simple study of the successful side and the lack of dialectical consideration make the study of metaphysics. (3) The theory is too fragmented and not systematic. Most of the existing studies start from a single dynamic factor of teenagers' campus basketball, such as social factor, institutional factor, and school factor. Although the research of these factors can reveal some superficial reasons for the confusion of teenagers' campus basketball development to a certain extent, it cannot solve the deep-seated contradictions in the development of Chinese campus basketball dynamic, so that the theory appears scattered, fragmented, and not systematic. (4) There are theoretical research gaps. The existing research on the development power of Chinese campus basketball is rare, and there is no in-depth research on the dynamic mechanism, so there is a large research space in this field.

## 3. Method

### 3.1. Based on Chan Algorithm

TOA/TDOA positioning model is one of the most commonly used high-precision positioning models. A certain signal (usually electromagnetic wave signal) is transmitted through the base station. When receiving the signal, the arrival time or arrival time difference of the signal is obtained through the time delay estimation algorithm, and then the distance from the target is obtained by multiplying the propagation speed of the signal. If the actual measured ti, *i* = 1,2,…,*N* obtained after time delay estimation is assumed, the distance measured value is *δi* = *c*ti, *i* = 1,2,…,*N*, where *c* = 299792458 m/*s* represents the speed of light [3].

Thus, the TOA positioning model of a single target can be obtained by establishing the distance equations between the base station and the target. Let Ri represent the measured distance between the *i*-th positioning base station and the positioning target, as shown in formula:

(1) $$\begin{array}{c} R_{i}=\delta_{i}=\sqrt{{\left(x_{i}-x_{0}\right)}^{2}+{\left(y_{i}-y_{0}\right)}^{2}},\;i=1,2,\ldots ,N. \end{array}$$

The position of the target to be located is *s*0 = (*x*0, *y*0), as shown in formula:

(2) $$\begin{array}{c} R_{i}^{2}={\left(x_{i}-x_{0}\right)}^{2}+{\left(y_{i}-y_{0}\right)}^{2}=K_{i}-2x_{i}x_{0}-2y_{i}y_{0}+x_{0}^{2}+y_{0}^{2}, \end{array}$$

where *Ki* = *xi*2 + *yi*2. Due to the existence of square term, the above formula becomes a nonlinear equation [4]. By making *R*02 = *x*02 + *y*02, the linear equation is as follows:

(3) $$\begin{array}{c} R_{i}^{2}-K_{i}=-2x_{i}x_{0}-2y_{i}y_{0}+R_{0}. \end{array}$$

Although *x*0, *y*0, and *R*0 are not independent of each other, the core idea of Chan algorithm is to adopt the two-step weighted least squares method (WLS). First assume that the two intermediate variables are independent of each other, linearize the nonlinear equation, use the weighted least squares to obtain their estimated value, and then consider the relationship between them, so that the target position can be solved. Thus,

(4) $$\begin{array}{c} h=\left[\begin{array}{c} R_{1}^{2}-K_{1}\\ R_{2}^{2}-K_{2}\\ \vdots \\ R_{N}^{2}-K_{N} \end{array}\right],\\ G_{a}=\left[\begin{array}{ccc} -2x_{1} & -2y_{1} & 1\\ -2x_{2} & -2y_{2} & 1\\ \vdots & \ddots & \vdots \\ -2x_{N} & -2y_{N} & 1 \end{array}\right],\\ Z_{a}=\left[\begin{array}{c} x\\ y\\ R \end{array}\right], \end{array}$$

where *x*, *y,* and *R* are the estimated values of *x*0, *y*0, and *R*0, respectively, as shown in formula:

(5) $$\begin{array}{c} R=x^{2}+y^{2}. \end{array}$$

The error vector of noise is defined as

(6) $$\begin{array}{c} \psi =h-G_{a}Z_{a}. \end{array}$$

Assuming that the system has a high signal-to-noise ratio, it can be considered that the measured values are Gaussian data; that is, they obey the approximate normal distribution. Since the noise vector *n* also obeys the approximate normal distribution, the vector statistical relationship about the error can be obtained as follows: as shown in formula:

(7) $$\begin{array}{c} \psi =2cBn+c^{2}n\cdot n, \end{array}$$

where *B* = diag {*r*1, *r*2,…, *rN*}, *r*1, *r*2,…, *rN* is the real distance between the positioning base station I and the positioning target. So BT = *B*, as shown in formula

(8) $$\begin{array}{c} R_{i}=r_{i}+cn_{i}. \end{array}$$

Since cni ≪ *r* holds in the actual application scenario, the tail term of (7) can be ignored and the error vector can be changed into a random vector [12]. The error vector can be written as follows:

(9) $$\begin{array}{c} \varphi =E\left(\psi \psi^{T}\right)\approx 4c^{2}BQB, \end{array}$$

where *Q* = diag {*σ*12, *σ*22,…, *σN*2} is the covariance matrix of the measured value. Assuming that each quantity in Za is independent of each other, it is obtained by weighted least squares, as shown in formula

(10) $$\begin{array}{c} Z_{a}={\left(G_{a}^{T}\varphi^{-1}G_{a}\right)}^{-1}G_{a}^{T}\varphi^{-1}h. \end{array}$$

Since there is the distance between the positioning target and the positioning base station in *B*, *ϕ* is an unknown quantity. Next, we have the problem of calculating *ϕ*. If the positioning target is far away from the positioning base station, *R*1 and *Ri* can be approximately considered to be equal. Therefore, when estimating *ψ*, the approximate replacement B of R1 I can be used, and *B* = diag {*r*1, *r*2,…, *rN*} is the true distance between the median base station I and the positioning target. Therefore, the approximate reduction of (10) can be as follows:

(11) $$\begin{array}{c} Z_{a}\approx {\left(G_{a}^{T}Q^{-1}G_{a}\right)}^{-1}G_{a}^{T}Q^{-1}h. \end{array}$$

If the positioning target is close to the positioning base station, an estimation solution can also be obtained by using the above formula. The approximate “real” distance between the positioning base station and the positioning target can be calculated by using the initial estimation solution and the coordinates of the positioning base station, so as to obtain the B matrix and then use (10) to obtain the first weighted least squares result [13]. Since the relationship between *x*, *y,* and *R* is not considered in the first weighted least squares, it will be considered in the second weighted least squares, so as to achieve higher positioning accuracy. Using the first estimated value, a set of error equations is constructed for the second estimation, as shown in formula

(12) $$\begin{array}{c} \left\{\begin{array}{c} Z_{1}=x_{0}+e_{1},\\ Z_{2}=x_{0}+e_{2},\\ Z_{3}=x_{0}+e_{3}, \end{array}\right. \end{array}$$

where *Zi* represents the *i*-th component in *Za* and *ei* represents the estimation error of *Za*. Define a new error vector as shown in formula:

(13) $$\begin{array}{c} \psi^{\prime }=h^{\prime }-G^{\prime }z^{\prime }, \end{array}$$

where

(14) $$\begin{array}{c} h^{\prime }=\left[\begin{array}{c} {\left(Z_{1}-X_{1}\right)}^{2}\\ {\left(Z_{2}-Y_{2}\right)}^{2}\\ Z_{3}^{2} \end{array}\right],\\ G^{\prime }=\left[\begin{array}{cc} 1 & 0\\ 0 & 1\\ 1 & 1 \end{array}\right],\\ z^{\prime }=\left[\begin{array}{c} {\left(x_{0}-X_{1}\right)}^{2}\\ {\left(y_{0}-Y_{1}\right)}^{2} \end{array}\right], \end{array}$$

where *S* = (*X*1, *Y*1) represents the known coordinates of base station 1, and the covariance matrix of *ψ*′ can be expressed as

(15) $$\begin{array}{c} \varphi^{\prime }=E\left(\psi^{\prime }\psi^{\prime T}\right)=4B^{\prime }\text{Cov}\left(Z\right)B^{\prime }. \end{array}$$

We have

(16) $$\begin{array}{c} B^{\prime }=\text{diag}\left\{x_{0}-X_{1},y_{0}-Y_{1},R_{0}\right\},\\ \text{Cov}\left(Z\right)=E\left(ee^{T}\right). \end{array}$$

Similarly, the previous method is used for estimation, and the result is as shown in formula

(17) $$\begin{array}{c} Z^{\prime }={\left(G^{\prime T}\varphi^{\prime -1}G^{\prime }\right)}^{-1}G^{\prime T}\varphi^{\prime }h^{\prime }. \end{array}$$

Finally, the final estimated position is obtained *Z* = ±Z′ + *S*_0_.

It can be seen from Chan algorithm that when the target is close to each base station, the first estimation also needs an estimated initial value to solve the initial solution estimation matrix. In real life, such as youth basketball scene, such a situation is very common [14].

### 3.2. Multivariate Taylor Algorithm

There are *N* base stations and *M* targets to be tested in the site. Because the traditional Taylor series expansion algorithm does not take into account the measured distance between the targets to be measured, it will lose some useful information, resulting in the loss of positioning accuracy.

The original Taylor algorithm only considers the distance relationship between the target to be tested and the base station, that is,

(18) $$\begin{array}{c} \left\{\begin{array}{c} R_{ij}=\sqrt{{\left(x_{1}-X_{j}\right)}^{2}+{\left(y_{i}-Y_{i}\right)}^{2}},\;i<j,\\ \vdots \\ R_{MN}=\sqrt{{\left(x_{M}-X_{N}\right)}^{2}+{\left(y_{M}-Y_{N}\right)}^{2}}, \end{array}\right., \end{array}$$

where *Ri*,*j* represents the measured distance between the target to be measured and the known base station [15]. In order to make the positioning more accurate, Taylor algorithm based on multivariate variables is proposed, and the measured distance between the targets to be measured is added to establish the equations, as shown in formula:

(19) $$\begin{array}{c} \left\{\begin{array}{c} R_{ij}^{\prime }=\sqrt{{\left(x_{i}-x_{j}\right)}^{2}+{\left(y_{i}-y_{j}\right)}^{2}},\;i<j,\\ \vdots \\ R_{M-1,M}^{\prime }=\sqrt{{\left(x_{M-1}-x_{M}\right)}^{2}+{\left(y_{M-1}-y_{M}\right)}^{2}}, \end{array}\right., \end{array}$$

where (*xi*, *yi*) represents the coordinate value of the target to be measured, (*Xi*, *Yi*) represents the coordinate value of the known base station, *R*′*i*,*j* represents the distance measurement value in the target to be measured, and *Ri*,*j* represents the distance measurement value between the target to be measured and the known base station.

After finishing, the positioning model is obtained, as shown in formula

(20) $$\begin{array}{c} h=G\Delta +E. \end{array}$$

Using the weighted least squares (WLS) method for (20), the estimation of Δ can be obtained as shown in formula (21).

Since the measured value may have delay errors caused by NLOS or multipath and the post-Taylor series expansion algorithm is sensitive to the initial value, it is necessary to discard the error data after obtaining the initial estimated value and before starting the Taylor algorithm [16]. See Figure 4.

A and B are base stations, *T* is the real target, *e* is the expectation of measurement error, and the equation of the circle is

(21) $$\begin{array}{c} R_{iA}=\sqrt{{\left(x_{i}-X_{A}\right)}^{2}+{\left(y_{i}-Y_{A}\right)}^{2}},\\ R_{i,B}=\sqrt{{\left(x_{i}-X_{B}\right)}^{2}+{\left(y_{i}-Y_{B}\right)}^{2}}. \end{array}$$

In theory, the distance measurement values of *A* and *B* are between the large circle radius and the small circle radius. Since an initial value has been obtained according to the Chan algorithm, it is substituted into the initial value to calculate the error of each base station from the initial value and calculate the cumulative distribution function to remove the error of more than 90%, which can not only improve the performance of a part, but also screen out some data [17].

### 3.3. Algorithm Flow

As shown in Figure 5, algorithm steps are as follows:

1. Randomly generate the initial solution *ω* and calculate the objective function *J* (*W*). The current number of iterations *k* = 0, and the current temperature *t*0 = *T*_max_, *r* ∈ (0, 1) is used to control the cooling annealing.
2. The disturbance generates a new solution *ω*′ and calculates the objective function *J* (*ω*′).
3. Calculate the increment Δ*J* = *J* (*ω*′)—*J* (*ω*).
4. If Δ*J* < 0, accept the new solution *ω* ← *ω*′, *k* ← *k* + 1 and reduce the temperature *tk* = rtk—1; otherwise, accept the new solution according to the Metropolis criterion; that is, accept the new solution with the probability *e*−Δ*J*/tk.
5. Judge whether the number of iterations has been reached. If not, continue with step 2.
6. Judge whether the termination conditions are met. The termination conditions are that the termination temperature is reached and the temperature is full [18].
7. If sufficient, output the final result. If not, reset the number of iterations *k* = 0 and reduce the initial temperature *t*0 = rtmax.
8. Get the initial value of coordinate estimation (*x*′, *y*′).
9. Use the initial value to calculate the matrix *B* in Chan algorithm, then substitute into (9) to calculate *ϕ* and then use (10) to calculate the first least squares solution *Za*.
10. Since the relationship between *x*, *y,* and *R* is not considered in the first least squares, it will be considered in the second least squares, so as to achieve higher positioning accuracy. Use (13)–(16) to find *Z*′ = (*G*′*Tφ*′-1*G*′)-1*G*′*Tφ*′*h*′.
11. Get the final estimated position. *Zi* = ±*Zi*′ + *S*_0_.
12. Calculate whether there is | | *Ri*, *B*—*Ri*, *A* |—RAB | > 4*σ*2 through the measured value. If there is, round off the large circle equation.
13. Carry out Taylor series expansion at the initial estimated values (*x*01, *y*01),…,(*x*0*M*, *y*0*M*) of the target to be measured, remove the components above the second order, and obtain the equations. After finishing, we get *h* = *G*Δ + *E*.
14. Using the weighted least square method (WLS), the estimation of ^Δ^ can be obtained: ^Δ^ = (GTQ-1*G*)-1GTQ-1*h*.
15. Repeat the calculation for many times until ^Δ^*xi* and ^Δ^*yi* are small enough to meet a set threshold *ε*。
16. Get the final result (*x*1, *y*1),…,(*xM*, *yM*).

It is assumed that the distance measurement error follows the exponential distribution of 10 m and the variance is *δ*2 = 1. See Figure 6.

Under other unchanged conditions, analyze the relationship between the variance of error and positioning accuracy: see Figure 7.

When *δ*2 = 0.5, repeat the test for 50 times to test the relationship between the positioning error distribution function and variance, as shown in Figure 8.

When the real target is at (60, 65) points, run the algorithm 20 times to obtain the location point distribution. See Figure 9.

When the distance measurement error follows the standard normal distribution with variance *δ*2 = 1: see Figure 10.

Increase the number of base stations to check the change of algorithm accuracy: see Figure 11.

Through the simulation analysis, it can be seen that the algorithm proposed in this paper has higher positioning accuracy when the channel conditions are not good enough and there are few base stations, but there are multiple targets to be measured. It is widely applicable in the real scene [19].

## 4. Experimental Results and Discussion

### 4.1. Experimental Results

In this paper, the recognition results and prediction results of the target detection system for the cultivation of the ring tone of juvenile basketball in the national fitness environment are presented. The accuracy of prediction refers to the ratio of predicting an athlete's movement to the real value (ground truth). It can be seen that the recognition and prediction accuracy of shooting action by this method is more than 85%. However, the accuracy of rebounding and passing recognition and prediction is low. The recognition accuracy and prediction accuracy of the test set are slightly lower than that of the effective set, which shows that the performance of the target detection system model in this paper can be further improved through more significant training examples [20].

According to the specific basketball movement, the corresponding actions in the target detection systemrebounding, shooting, and passing—are reconstructed based on the key points of human body. The method proposed in this paper can help basketball players better adapt to various training methods and tactical training to a certain extent and quickly improve their performance. Linear regression analysis is carried out on the automatic scoring of the target detection system in rebounding, shooting, passing, and fine motion evaluation (the algorithm proposed in this paper) and the traditional manual scoring to study their correlation. Each point in the figure represents the result of a test, the abscissa represents the evaluation score obtained by the automatic evaluation algorithm, and the ordinate represents the real value evaluated by the traditional training method. It can be seen that the score of the automatic evaluation algorithm is linear with that of the traditional training method. Compared with the traditional training method, the fine motion obtained by the target detection system in this paper has certain advantages and can bring better teaching effect. This combination of explanation and demonstration can greatly stimulate athletes' senses and make them have a deeper memory and a deeper understanding of technology. See Figures 12–16.

In addition, the traditional model generally cannot recover some arm posture features of basketball, such as severe occlusion, high moving speed, sudden direction change, and a large number of physical confrontation between players. These features challenge the accuracy of the detection efficiency of individual players and teams. Therefore, after detecting the players, the target detection and fine positioning method proposed in this paper cuts the area where the detected players are located and divides five motion channels through the statistics of arm posture characteristics to get the characteristics of arm posture distribution, so as to identify the subordinate relationship of basketball playing method and obtain a more fine detection and fine positioning method [21]. Because the prior conditions of unified arm posture are obtained, this method can classify the subordinate relationship of basketball playing without additional annotation during the construction of data set and can more accurately identify the technical skills of basketball far mobilization. Compared with the detection accuracy in the models of integrated channel features (ICF), fast recursive convolution neural network (RCNN), and single shot multibox detector (SSD 512), it can be seen that the accuracy of this method is 95.6% in all algorithms, which shows that the target detection system designed in this paper is effective. See Figure 17.

### 4.2. Using Physical Exercise to Improve the Mental Health of Adolescents

1. *The Cultivation of Emotional Cognition and Personality through Physical Exercise*
2. Personality refers to the internal tendency and psychological characteristics of an individual's behavior in social adaptation to people, things, and themselves. Psychosomatic organization, wholeness, stability, uniqueness, and sociality are the basic characteristics of personality. Physical exercise can allow young people to analyze the differences between themselves and others in such a so-called social adaptation process, learn from the strong in terms of ability, temperament, character, needs, etc., and constantly improve their shortcomings and allow themselves to grow. It is more comprehensive, and at the same time, it can retain its own personality characteristics and finally form the so-called personality charm. In this process, there will always be people-to-people communication, whether it is friendly communication or communication with other emotions, which can enrich the personal emotions and self-cognition level of teenagers. Knowledge decline is slowed down, individuals develop a more active way of releasing stress, and desired personality traits are maintained. Only then can it be called the complete cultivation of a person.
3. *The Cultivation of Willpower through Physical Exercise*
4. Willpower refers to the quality of a person who consciously determines the purpose, controls and adjusts his actions according to the purpose, overcomes various difficulties, and thus achieves the purpose. When teens are adept at harnessing this beneficial force, determination develops. And the determination of a person shows that willpower is at work. Faced with the huge pressure of learning and social life in today's society, young people need to cultivate a strong will quality, which is also one of their essential qualities on the road to success. There are many situations in physical exercise that can cultivate good willpower. For example, when the score is behind, you should make tactical and technical changes in time to try to reverse the situation and rewrite the score; in the case of minor injuries, adjust your skills reasonably and appropriately. The movement and the way of exertion can complete the whole physical exercise process.

## 5. Conclusion

This paper presents a method to develop the ring tone of juvenile basketball in the national fitness environment. First of all, after analysis and discussion, it is clear that physical exercise has a positive effect on the mental health of young people, can effectively regulate the emotions of young students, let the body get rid of the subhealth state as much as possible, and get physical and mental benefits. Improve, so that you can better devote yourself to high-intensity and high-load learning activities. From another aspect, it can cultivate the self-confidence of young people in social activities, dare to communicate with others actively and understand the importance of teamwork. The specific content of this method is based on the Chan algorithm. When the target is close to each base station, the first estimation also needs an estimated initial value to solve the initial solution matrix. In real life, such as youth basketball scene, this situation is very common, and under the simulation analysis of multivariate Taylor algorithm, the proposed algorithm has higher positioning accuracy when the channel conditions are not good enough and there are few base stations, but there are multiple targets to be measured, so it has wide applicability in real scene. To prove that this method can solve the problem of cultivating the ring tone of juvenile basketball in the national fitness environment, the specific performance is as follows: among all the algorithms for cultivating the ring tone of juvenile basketball, the accuracy rate is the highest, reaching 95.6%. In the future national fitness environment, it will be more and more important to develop the environmental tonality of juvenile basketball. It is believed that Chan algorithm and multivariate Taylor algorithm will be widely used in different scenarios in the near future.

## Figures and Tables

**Figure 1:** The role of national fitness behavior and effect.

**Figure 2:** Social movement mechanism system.

**Figure 3:** Youth campus basketball power difficulty.

**Figure 4:** Range of theoretical measured values.

**Figure 5:** Algorithm flow chart.

**Figure 6:** Error analysis of different algorithms.

**Figure 7:** Comparison of positioning errors of different algorithms.

**Figure 8:** Relationship between cumulative distribution and measurement error variance.

**Figure 9:** Location point distribution of algorithm.

**Figure 10:** Error analysis of different algorithms.

**Figure 11:** Relationship between the number of base stations and positioning error.

**Figure 12:** Comparison between recognition results and prediction results of coordination of juvenile basketball players.

**Figure 13:** Backboard prediction results.

**Figure 14:** Shooting prediction results.

**Figure 15:** Pass prediction results.

**Figure 16:** Fine motion prediction results.

**Figure 17:** Comparison between the method in this paper and other methods.

## Data Availability

The labeled data set used to support the findings of this study is available from the corresponding author upon request.
